RETRACTED

# Evaluation of Critical Factors of Postoperative Arrhythmia and Preventive Measures of Deep Venous Thrombosis

**DOI:** 10.1155/2021/6103092

**Published:** 2021-11-24

**Authors:** Boheng Liu, Mingbo Wang, Jiawei Dong, Hao Wang, Ziqiang Tian

**Affiliations:** Department of Thoracic Surgery, The Fourth Hospital of Hebei Medical University, No. 169 Tianshan Street, Economic and Technological Development District, Shijiazhuang 050035, Hebei, China

## Abstract

The study focused on the risk factors of postoperative arrhythmia and lung infection and the preventive effects of targeted low-molecular-weight heparin (LMWH) on the occurrence of deep venous thrombosis (DVT) in patients with esophageal/cardia cancer. In this article, 82 patients who were pathologically diagnosed with esophageal/cardia cancer and underwent surgical treatment were selected as the research subjects. According to the different preoperative treatment methods, the patients were divided into the control group (without anticoagulant drugs before the operation, 44 cases) and the anticoagulation group (anticoagulant drugs were administered before the operation, 38 cases), and they were compared for basic clinical indicators and disease history. Logistic regression analysis was performed to analyze the risk factors of adverse events, and the Wells and Autar scale scores were calculated. Different groups were compared for the operation time, blood loss, and postoperative drainage volume during the operation. D-dimer was detected on the first 1, 3, 5, and 7 days after the operation, and the lower extremity venous color Doppler ultrasound was performed on the 1st and 7th days after the operation. The results showed that age ≥65 years, abnormal preoperative ECG, preoperative coronary heart disease (CHD), preoperative chronic obstructive pulmonary disease (COPD), operative time ≥4 h, and preoperative blood sodium <4.04.0 mmol/L were all risk factors for postoperative arrhythmia. Age, preoperative diabetes mellitus, preoperative COPD, length of hospital stay, and FEV1 were all risk factors for postoperative lung infections. In the control group and anticoagulation group, 11 cases (13.41%) and 5 cases (16.10%) had lower extremity DVT, respectively. The incidence of lower extremity DVT was lower in the anticoagulation group than in the control group (*P* < 0.01). It suggested that age, preoperative disease history, hospital stay, and operation time were risk factors for postoperative adverse events in patients with esophageal/cardia cancer. The targeted anticoagulant LMWH has a significant preventive effect on the occurrence of lower extremity DVT in patients with esophageal/cardia cancer, providing an effective reference for the prognosis and prevention of esophageal/cardia cancer.

RETRACTED

## 1. Introduction

Esophageal/cardia cancer is a common malignant tumor of the digestive tract. According to statistics, the incidence of esophageal/cardia cancer is the eighth among all malignant tumors in the world, and the mortality rate ranks sixth. The number of new cases of esophageal/cardia cancer is about 456,000 every year, of which about 300,000 die every year, 80% of whom are distributed in developing countries [1]. The incidence of esophageal/cardia cancer in China is high, accounting for about 50% of all cases in the world. The incidence of esophageal/cardia cancer ranks fifth among all malignant tumors in China, but its mortality rate is second only to lung, stomach, and liver cancer. It is estimated that the incidence of esophageal cancer in China will increase by 140% in the next decade [2]. Since most esophageal/cardia tumors are adenocarcinomas, and adenocarcinomas are less sensitive to chemotherapy drugs and radiation, and thus, radiotherapy and chemotherapy are not effective for esophageal/cardia cancer. At present, surgical methods are mainly used to treat esophageal/cardia cancer [3]. However, after treatment, the postoperative survival rate is low and the quality of life is poor, accompanied by postoperative complications [4]. The currently used surgical methods include radical resection of cardia cancer through the thoracic incision, radical resection of cardia cancer through an abdominal incision, and radical resection of cardia cancer through the combined thoracoabdominal incision. The radical resection of cardia cancer through thoracic incision has a large incision wound that is beneficial to the thorough removal of the mediastinum and intrathoracic lymph nodes, but it increases the incidence of complications in heart and lung systems [5]. Radical resection of cardia cancer with abdominal incision has a small wound area, which reduces the occurrence of complications of the heart, lung, breathing, and circulatory systems, but it fails to completely remove the mediastinal lymph nodes [6]. Radical resection of cardia cancer through combined thoracoabdominal incision significantly increases the incidence of postoperative complications such as lung infection and arrhythmia in patients resulting from its large incision and long operation time [7]. Therefore, early prevention, early detection, and timely treatment of complications will play an important role in the postoperative recovery of patients with esophageal/cardia cancer. However, there are few studies on risk factors related to adverse events after esophageal/cardia cancer surgery.

RETRACTED

Deep venous thrombosis (DVT) refers to venous tube obstruction arising from abnormal coagulation of the body's venous blood, which causes the patient to have limb pain, swelling, and other clinical symptoms [8]. Surgical treatment of esophageal/cardia cancer can easily cause DVT of the lower limbs after surgery. If not treated in time, it can also lead to the occurrence of the postoperative DVT syndrome in severe cases [9]. At present, color Doppler ultrasound, spiral CT vein imaging, MRI vein imaging, venography, and C-reactive protein and D-dimer are often used for diagnosis [10]. Patients with postoperative lower limb DVT mainly use mechanical therapy, anticoagulation therapy, surgical treatment, and thrombolytic therapy. At the same time, adequate postoperative hydration, intravenous nutritional support, analgesia, use of anticoagulant drugs, and intermittent airbag compression of the affected limb can also be used to prevent the occurrence of postoperative DVT in the lower limbs [11]. The targeted anticoagulant drug low-molecular-weight heparin can be combined with antithrombinl to inhibit the activity of coagulation factor Xa and reduce the occurrence of bleeding and thrombocytopenia. The current research results show that the use of 4,000∼6,000 u targeted anticoagulant LMWH can effectively alleviate the clinical symptoms of patients with postoperative lower extremity DVT [12]. Nevertheless, there are few reports on whether the targeted anticoagulant LMWH can effectively prevent the occurrence of DVT in the lower limbs of patients with esophageal/cardia cancer.

Above all, there are many risk factors for adverse events after esophageal/cardia cancer. It is not known whether the targeted anticoagulant LMWH can effectively prevent the occurrence of DVT in the lower limbs of patients with esophageal/cardia cancer. Therefore, 82 cases of patients diagnosed with esophageal/cardia cancer pathologically were selected as research subjects in this study to analyze the risk factors of postoperative adverse events in patients with esophageal/cardia cancer and further explore the preventive and therapeutic effects of LMWH, a targeted anticoagulant drug, on DVT of lower limbs. The study was intended to provide a reference for the prognosis of patients with esophageal/cardia cancer and the prevention and treatment of DVT in lower limbs after the operation.

## 2. Materials and Methods

### 2.1. Research Subjects and Grouping

From January 2019 to December 2020, 82 patients who were pathologically diagnosed with esophageal/cardia cancer in the Gastroenterology Department of The Fourth Hospital of Hebei Medical University and were treated with surgery were selected as the research subjects, including 59 males and 23 females, ranging in age from 37 to 85 years, with an average age of (61.74 ± 9.65) years. The inclusion criteria for this study were as follows: (1) adults older than 18 years; (2) patients with primary esophageal/cardia tumors and accepted surgical treatment; (3) patients with no history of drug allergy; (4) patients with complete clinical data; (5) coagulation function was normal before surgery; and (6) patients with no history of venous thrombosis or embolism. Exclusion criteria were as follows: (1) patients with severe heart, liver, kidney, and other system diseases; (2) patients with a history of other malignant tumors; and (3) patients with surgical contraindications. The criteria for rejection were as follows: (1) patients who died during clinical observation; (2) patients not completing the treatment due to various reasons; and (3) patients who used other drugs that had an impact on the results of this study. According to different preoperative treatments, patients were divided into control group (no anticoagulant drugs before the operation) and anticoagulant group (anticoagulant drugs were given before the operation). There were 44 cases in the control group and 38 cases in the anticoagulant group. The patients were further divided into event group and no event group according to whether there were adverse events after the operation. The trial process of this study has been approved by the ethics committee of The Fourth Hospital of Hebei Medical University, and all subjects included in the study have signed an informed consent form.

RETRACTED

### 2.2. Treatment Methods for Patients with Esophageal/Cardia Cancer

After admission, all patients were required to undergo ultrasound, electrocardiogram, and color Doppler ultrasound examinations to detect blood coagulation function and life indicators. Additionally, preoperative ultrasound, gastroscopy pathology, and color Doppler ultrasound examination of the lower limb veins were performed. Before the operation, the patients were forbidden to smoke for two weeks, and the patients with respiratory tract infections were treated with anti-infection and nebulization methods before treatment. Sodium phosphate salt solution was used to clean the gastrointestinal tract 24 hours before surgery. The patient was required to fast for 12 hours, and drinking was forbidden for more than 4 hours. Antibiotics were given 2 h before surgery to prevent postoperative wound infection. Patients in the anticoagulation group were injected subcutaneously with low-molecular-weight heparin calcium-targeted anticoagulants (Subilin, Tianjin GlaxoSmithKline Co. Ltd.) 24 hours and 12 hours before surgery at a dose of 0.004 mL/kg, and patients in the control group accepted conventional treatment. All patients were anesthetized with single tracheal intubation and treated using left thoracic aortic arch gastroesophageal anastomosis; left thoracic aortic arch gastroesophageal anastomosis; left thoracic and neck two-incision gastroesophageal neck anastomosis; three-incision gastroesophageal neck anastomosis on right chest, abdomen, and neck; and left chest and abdomen two-incision total gastrectomy and jejunal esophagus anastomosis to completely remove the tumor and the regional lymph nodes. After the operation, the patient was monitored by ECG, accompanied by oxygen inhalation and calorie supplementation. The energy was supplemented at 25–35 kcal/kg/d, and vitamins and trace elements were appropriately given. Antibiotics were used to prevent infections of the lungs, abdominal cavity, and surgical incisions after 1 to 2 days, intravenous analgesia was given for 2 to 3 days, and oxygen masks were nebulized to assist in expectoration.

RETRACTED

### 2.3. Diagnostic Criteria and Evaluation Methods of DVT of Lower Extremities

The diagnosis was made according to the diagnostic criteria for DVT of the lower limbs established by the Vascular Surgery Group of the Chinese Medical Association Surgery Branch, and the diagnosis was confirmed by color Doppler ultrasound.

All patients were assessed for the risk of DVT of the lower extremities by the Wells clinical assessment scale and Autar scale before the operation and on the 1st and 7th day after the operation. The Wells lower extremity DVT risk assessment scale has 9 items. According to the total score of each item, the risk of DVT in lower extremities is divided into three levels, with ≥3 points indicating high risk, 1∼2 points indicating intermediate risk, and ≤0 points indicating low risk [13]. The Autar lower extremity DVT risk assessment scale covers 7 items including the patient's age, trauma risk, high-risk diseases, and surgery. Based on the total score of each item, the risk of DVT in lower extremities is divided into three levels, with ≥15 points indicating high risk, 11–14 points indicating intermediate risk, and ≤10 points indicating low risk [14].

### 2.4. Observation Index

The basic information of the patient was recorded, including the age, body mass index (BMI), disease history, and other basic clinical treatments. The Wells and Autar scale scores were calculated before and after surgery. The blood routine and coagulation function indexes before surgery were tested and different groups of patients were compared for the operation time, blood loss, and postoperative drainage volume during the operation. D-dimer was detected on the 1st, 3rd, 5th, and 7th days after the operation, and color Doppler ultrasound examination was performed to detect the lower extremities on the 1st and 7th days after the operation. Postoperative lung infection and arrhythmia were regarded as adverse events in this study.

RETRACTED

### 2.5. Statistical Analysis

SPSS21.0 was used to process the data. Normally distributed measurement data were expressed as mean ± standard deviation $\left(\bar{x}\pm s\right)$, and the independent sample *t*-test was used. The chi-square test was used to count data. Logistic regression was used to analyze the occurrence of adverse events in patients with esophageal/cardia cancer. The difference was statistically significant with *P* < 0.05.

## 3. Results and Discussion

### 3.1. Risk Factors for Postoperative Arrhythmia

A total of 13 patients in all subjects included in this study had arrhythmia after surgery, accounting for 15.85%. The index differences between patients with arrhythmia and normal patients were analyzed (Figure 1). Of the 13 patients with arrhythmia, 11 patients were older than 65 years old, accounting for 84.62%, higher than the proportion in the normal group where there were 28 cases older than 65 years old, accounting for 40.58% (*P* < 0.05). There were 8 (61.54%) and 20 (28.99%) patients with abnormal ECG before the operation in the arrhythmia group and normal group, respectively. The proportion of patients with abnormal ECG before the operation in the arrhythmia group was higher than the normal group (*P* < 0.05). In the arrhythmia group, there were 3 patients (23.08%) with coronary heart disease (CHD) and 3 patients (23.08%) with chronic obstructive pulmonary disease (COPD) before the operation. In the normal group, there were 1 patient (1.45%) with CHD and 3 patients (4.35%) with COPD before the operation. The proportion of patients with preoperative CHD in the normal group was lower than the abnormal group (*P* < 0.001). The proportion of patients with preoperative COPD in the arrhythmia group was higher than that of the normal group (*P* < 0.01). In the arrhythmia group, there were 7 cases (53.84%) with operation time ≥4 h, and in the normal group, there were 12 cases (17.39%). The proportion of patients with operation time ≥4 h in the arrhythmia group was higher than that in the normal group (*P* < 0.01). In the arrhythmia group, there were 5 patients (38.46%) with preoperative serum potassium <4.0 mmol/L, and the proportion was higher than the normal group (13 patients (18.84%); (*P* < 0.05).

Logistic multivariate regression analysis was performed to analyze the risk factors of the adverse events of arrhythmia. It was noted that age ≥65 years old, preoperative ECG abnormality, preoperative CHD, preoperative COPD, surgery time ≥4 h, and preoperative serum potassium <4.0 mmol/L were risk factors for postoperative arrhythmia (Table 1).

RETRACTED

### 3.2. Analysis of Risk Factors of Postoperative Lung Infection

The lung infection and noninfection groups were compared for indexes such as albumin (Alb), platelet count (PLT), maximum mid-expiratory flow (MMEF), and length of stay. The average age was (65.92 ± 9.78) years and (60.77 ± 10.03) years, respectively (*P* < 0.01). The blood loss, Alb, and PLT of patients in the infection group were (185.48 ± 19.11) mL, (45.17 ± 14.45) g/L, and (228.99 ± 15.06) × 10^9^/L, respectively, showing a difference versus the noninfection group (*P* > 0.05). The BMI of patients with lung infections was (23.16 ± 2.28) kg/m^2^, higher than the average BMI of patients in the noninfection group ((21.58 ± 2.09) kg/m^2^; (*P* < 0.01); Figure 2(a)). There was no significant difference in the number of lymph nodes, operation time, and forced vital capacity (FVC) between the two groups (*P* > 0.05). The hospital stay, MMEF, and forced expiratory volume in one second (FEV1) of patients in the infection group were (13.29 ± 1.92) d, (3.47 ± 0.93), and (3.61 ± 0.52) L, respectively, and those in the noninfection group were (9.94 ± 1.87) d, (3.14 ± 0.82), and (0.87 ± 0.51) L, respectively. Hence, *P* < 0.01 was for the hospital stay and FEV1 between the two groups. The MMEF value of the noninfection group was lower than that of the infection group ((*P* < 0.05); Figure 2(b)).

A total of 15 patients in all subjects included in this study developed a pulmonary infection after surgery, which accounted for 18.29%. Next, the two groups were compared for the preoperative history of diseases and the proportion of different pathological types (Figure 3). The number of patients in the infection group with diabetes, COPD, and CHD before surgery was 4 cases (26.67%), 3 cases (20.00%), and 14 cases (6.67%). In the noninfection group, there were 2 cases (2.99%), 3 cases (4.48%), and 3 cases (4.48%) with diabetes, COPD, and CHD before the operation. In the infection group, the proportion of patients with diabetes before the operation was higher (*P* < 0.001), and the proportion of patients with COPD was higher (*P* < 0.01). There was no significant difference in the proportion of patients with CHD, smoking history, adenocarcinoma, and squamous cell carcinoma before the operation between the two groups (*P* > 0.05).

Logistic multivariate regression analysis was used to analyze the risk factors for adverse events of lung infection. It was noted that age, preoperative diabetes, preoperative COPD, length of hospital stay, and FEV1 were all postoperative risk factors for a lung infection (Table 2).

RETRACTED

### 3.3. Comparison of Basic Information of the Two Groups of Patients

The control group and the anticoagulation group were compared for the indexes such as age, sex ratio, BMI, and pathological types. The differences in basic data of the two groups, such as age, sex ratio, and pathological types, were not statistically significant (*P* > 0.05). The average BMI of the control group was (23.87 ± 3.32) kg/m^2^, higher than the anticoagulation group ((22.95 ± 3.19) kg/m^2^; Table 3).

### 3.4. Postoperative Complications in the Two Groups

The postoperative complications of the two groups of patients were counted, and the results were shown in Figure 4. In the control group, there were 1 case (2.27%), 2 cases (4.55%), 1 case (2.27%), 3 cases (6.82%), 8 cases (18.18%), 2 cases (4.55%), 2 cases (4.55%), 3 cases (6.82)%), 1 case (2.27%), and 7 cases (15.91%) with anastomotic leakage, anastomotic stenosis, gastric stump fistula, thoracic-gastric syndrome, pulmonary complications, cardiovascular complications, gastric emptying disorders, respiratory failure, incision infection, and arrhythmia, respectively; in the anticoagulation group, there were 1 case (2.63%), 3 cases (7.89%), 1 case (2.63%), 3 cases (7.89%), 7 cases (18.42%), 2 cases (5.26%), 1 case (2.63%), 2 cases (5.26%), 1 case (2.63%), and 6 cases (15.79%) with anastomotic leakage, anastomotic stenosis, gastric stump fistula, thoracic and stomach syndrome, pulmonary complications, cardiovascular complications, gastric emptying disorder, respiratory failure, incision infection, and arrhythmia, respectively. There was no significant difference in the proportion of patients with different postoperative complications between the two groups (*P* > 0.05).

### 3.5. Statistics of Preoperative Complications of the Two Groups of Patients

The control group and the anticoagulation group were compared for the preoperative history of hypertension, diabetes, CHD, and COPD. The results are shown in Figure 5. In the control group, there were 5 cases (11.36%), 3 cases (6.82%), 2 cases (4.55%), and 3 cases (6.82%) with hypertension, diabetes, CHD, and COPD, respectively; in the anticoagulant group, there were 4 cases (10.53%), 3 cases (7.89%), 2 cases (5.26%), and 3 cases (7.89%) with blood pressure, diabetes, CHD, and COPD, respectively. There was no significant difference in the proportion of patients with hypertension, diabetes, CHD, and COPD before the operation between the two groups (*P* > 0.05).

### 3.6. Analysis of the Proportion of Patients with Different Surgical Methods in the Two Groups

All subjects included in this study were treated with surgical methods, and the proportion of different surgical methods was analyzed (Figure 6). In the control group, the left thoracic aortic arch gastroesophageal anastomosis; the left thoracic aortic arch gastroesophageal anastomosis; the left thoracic and neck two-incision gastroesophageal neck anastomosis; three-incision gastroesophageal neck anastomosis on the right chest, abdomen, and neck; and left chest and abdomen two-incision total gastrectomy and jejunal esophagus anastomosis were performed in 19 cases (43.18%), 13 cases (29.55%), 7 cases (15.91%), 4 cases (9.09%), and 1 case (2.27%), respectively; in the anticoagulation group, the corresponding number was 17 cases (44.74%), 11 cases (28.95%), 6 cases (15.79%), 3 cases (7.89%), and 1 case (2.63%), respectively. There was no statistical difference in the proportion of different surgical methods between the two groups (*P* > 0.05).

RETRACTED

### 3.7. Comparison of Surgical Indicators between the Two Groups

The two groups were compared for the operation anesthesia time, operation time, intraoperative blood loss, intraoperative fluid replenishment, and postoperative drainage volume (Figure 7). There was no statistically significant difference between the two groups in operative anesthesia time, operation time, intraoperative blood loss, intraoperative fluid replenishment, and postoperative drainage volume.

### 3.8. Incidence of DVT in Lower Extremities of the Two Groups of Patients before and after Surgery

The incidence of DVT in the lower extremities of the two groups of patients after surgery was analyzed (Figure 8). A total of 11 patients (13.41%) in the control group had DVT in the lower extremities after surgery, and only 5 patients (6.10%) in the anticoagulation group had DVT in the lower extremities. The incidence of DVT in the lower limbs of the anticoagulation group was significantly lower than that of the control group (*P* < 0.01).

### 3.9. Analysis of Color Doppler Ultrasound Results of Lower Extremity Vein in Two Groups of Patients

Doppler ultrasound was performed to detect postoperative lower extremity veins. Normal lower extremity ultrasound showed no echo and good sound penetration in the cavity (Figure 9(a)). The lumen was clearly displayed, with thickened veins, smooth inner walls, and good continuity (Figure 9(b)). Ultrasound Doppler venous blood flow chart showed that the blood flow signal was full and continuous (Figure 9(c)). After surgery, patients with DVT in the lower extremities showed solid echo fills with varying intensities in the ultrasound cavity (Figure 9(d)). Color Doppler ultrasound showed a filling defect at the thrombus (Figure 9(e)), and the venous blood flow chart showed no blood flow signal in the cavity (Figure 9(f)).

RETRACTED

### 3.10. Risk Assessment Scale for Lower Extremity DVT of the Two Groups of Patients before and after the Operation

The Wells clinical assessment scale and Autar scale were used to assess the risk of DVT in the lower extremities of the two groups of patients before surgery and on the 1st and 7th days after the surgery (Figure 10). Before surgery, there was no statistical difference between the control group and the anticoagulation group in the risk distribution. On the 1st day after the surgery, the proportion of high-risk and intermediate-risk patients in the control group showed an increase trend, while the anticoagulation group showed a downward trend, and the proportion of intermediate-risk patients between the two groups was statistically different (*P* < 0.05). On the 7th day after the surgery, the proportion of high-risk patients in the control group was higher (*P* < 0.001); the proportion of intermediate-risk patients in the control group was higher (*P* < 0.01); and the proportion of low-risk patients in the control group was lower (*P* < 0.05).

### 3.11. Comparison of D-Dimer Results between Two Groups of Patients

The D-dimer values of the two groups of patients before the operation, at 1 d, 3 d, 5 d, and 7 d after the operation were analyzed (Figure 11). The D-dimer values of the two groups of patients before the operation were (2351.28 ± 226.47) ng/L and (2179.93 ± 421.99) ng/L, respectively, *P* > 0.05. After surgery, the D-dimer values of the two groups both showed an upward trend. The D-dimer in the anticoagulation group was lower than the control group at 5 days after the operation (*P* < 0.05), and D-dimer in the anticoagulation group was lower than the control group at 7 days after the operation (*P* < 0.01).

## 4. Discussion

Arrhythmia and lung infections are common adverse events in patients with esophageal/cardia cancer [15]. For patients with esophageal/cardia cancer, the surgical treatment causes physiological and pathological changes in the respiratory and circulatory systems of the body, which increases the incidence of arrhythmia [16]. Arrhythmia affects the patient's cardiac output and circulatory function, leading to hypotension and cardiac arrest [17]. This study mainly analyzed the occurrence of arrhythmia and lung infection adverse events and their risk factors in patients with esophageal/cardia cancer. The results found that a total of 13 patients (15.85%) had arrhythmia after surgery. Gawinecka et al. [18] found that the incidence of postoperative arrhythmia in patients with esophageal/cardia cancer was 16.83%, in line with the results of the study. The results of the study showed that age ≥65 years, abnormal preoperative ECG, preoperative combined CHD, preoperative combined COPD, preoperative time ≥4 h, and preoperative serum potassium <4.0 mmol/L were all risk factors for postoperative arrhythmia. Tonnsen et al. [19] pointed out that the incidence of postoperative arrhythmia in elderly patients with esophageal cancer was increased (*P* < 0.01), consistent with the results of the study. The influence of old age on arrhythmia may be due to the gradual decrease in the density of sinus node cells and nerve fiber of the cardiac conduction bundle, which in turn increases the incidence of arrhythmia [20]. The long-term insufficient blood supply of the body's coronary arteries causes the proliferation of myocardial fibers, leading to CHD [21]. In patients with esophageal/cardia cancer, surgical anesthetics pull and squeeze the heart, lung, and other internal organs during the surgical process, causing coronary artery spasm, which can induce postoperative arrhythmia [22]. Preoperative ECG abnormality is one of the risk factors for postoperative arrhythmia, indicating that there is a certain correlation between the preoperative ECG abnormality and the occurrence of postoperative arrhythmia. This is because patients with abnormal ECGs mostly have myocardial autonomic cells or conduction abnormalities. They suffer from cardiopulmonary compression during surgery, which reduces lung ventilation function and myocardial oxygen utilization and ultimately leads to postoperative arrhythmia [23]. The myocardium of patients with COPD before surgery is more sensitive to hypoxia, which increases the incidence of postoperative arrhythmia. Studies have pointed out that the respiratory function and bronchial mucosal clearance of COPD patients are abnormal, and the postoperative pain at the incision limits breathing and expectoration, which imbalances the airway ventilation/blood flow ratio, leading to hypoxemia and at the same time increasing the occurrence of arrhythmia [24]. de Araujo Motta et al. [25] pointed out that the incidence of postoperative arrhythmia in patients with preoperative COPD increased by 3 times compared with normal patients. The results in this study showed that preoperative serum potassium <4.0 mmol/L was one of the risk factors for postoperative arrhythmia. The reason is that patients with esophageal/cardia cancer cannot eat normally before surgery for a long time, leading to varying degrees of malnutrition. After surgery, continuous gastrointestinal decompression will cause gastrointestinal potassium and magnesium and other water and electrolytes to be lost, leading to changes in cardiac function and increasing the incidence of the psychological disorder [26]. Hypokalemic esophageal/cardia cancer patients should be given a certain amount of potassium to reduce the incidence of arrhythmia.

RETRACTED

Current research results show that the incidence of postoperative lung infection in patients with esophageal/cardia cancer is between 7.3% and 50% [27], and the mortality rate is 10% to 40% [28]. The results of this study found that a total of 15 patients had lung infections after surgery, which accounted for 18.29%. This was aligned with the results of most current studies. The results in the study showed that age, preoperative diabetes, preoperative COPD, length of hospital stay, and FEV1 were all risk factors for a postoperative lung infection. Various body functions and organs of elderly patients tend to be aging. At the same time, the body's immunity and resistance are reduced, which reduces the patient's lung ventilation function and diffusion function and ultimately increases the incidence of lung diseases. Some reports have pointed out that patients with esophageal/cardia cancer older than 70 years have a significantly increased risk of a lung infection after surgery (*P* < 0.05) [29]. Esophageal/cardia cancer patients with diabetes mellitus have reduced body resistance and immune function, and as well as lung tissue resistance, which increases the risk of lung diseases. At the same time, long-term diabetes increases the body's glycosylated hemoglobin, reduces the release of oxygen, and ultimately induces hypoxemia, which leads to insufficient oxygen supply to the lung tissue, weakens the lung surfactant, and increases the occurrence of lung inflammation [30]. The operation time is related to the occurrence of postoperative lung infections in patients with esophageal/cardia cancer. The prolonged operation time leads to prolonged anesthesia time. Prolonged mechanical ventilation aggravates lung tissue compression, leading to postoperative pulmonary edema and hypoxemia [31]. Studies have pointed out that mechanical ventilation time >3 h will cause histopathological damage of the collapsed lung and increase the incidence of pneumonia [32]. Patients with preoperative COPD are mostly in a chronic hypoxic state. Various factors, such as surgical trauma, increased intraoperative blood loss and postoperative pain, reduced the patient's lung function, and increased the incidence of postoperative pulmonary infections [33]. If the patient has been hospitalized for a long time, the increase of drug-resistant bacteria in the ward increases the incidence of postoperative lung infections as a result of exposing the body to the medical environment for a long time. Seese et al. [34] pointed out that when the lung function index FEV1% < 50%, the incidence of lung infections increased significantly.

RETRACTED

DVT of the lower limbs is a common serious complication of surgery. In severe cases, it can cause pulmonary embolism, which directly affects the patient's treatment effect and quality of life. Under normal physiological conditions, the body's blood coagulation factors and anticoagulant substances are in a dynamic equilibrium state. The operation of thoracic surgery restricts the movement of the patient's lower limbs and the use of anesthetics during the operation increases the risk of postoperative DVT [35]. The targeted anticoagulant drug, low-molecular-weight heparin, can be combined with antithrombin to regulate coagulation factor Xa. Because of its good targeting, it is widely used in the treatment of DVT [36]. In the study, it was applied to prevent DVT in patients with esophageal/cardia cancer after surgery. The results found that the incidence of DVT in the lower extremities of patients in the anticoagulation group was significantly lower than that in the control group (*P* < 0.01). On the 7th day after the surgery, the proportion of high-risk patients in the control group was higher (*P* < 0.001); the proportion of intermediate-risk patients in the control group was higher (*P* < 0.01); and the proportion of low-risk patients in the control group was lower (*P* < 0.05). D-dimer in *the* anticoagulation group was lower than the control group at 5 days after the operation (*P* < 0.05), and D-dimer in the anticoagulation group was significantly lower than the control group at 7 days after the operation (*P* < 0.01). The occurrence of DVT in the lower limbs is related to intraoperative venous intima injury and blood flow stasis, which increase the level of procoagulant factors and impair the fibrinolytic mechanism [37]. D-dimer is a fibrin degradation product, and its concentration can be significantly increased in patients with acute thrombosis [38]. The results of this study suggested that the postoperative D-dimer values of the anticoagulation group and the control group were higher than those before the operation, and the reason is that the surgical trauma increases the body's D-dimer value. It indicates that the LMWH can effectively reduce the incidence of lower extremity DVT in patients with esophageal/cardia cancer.

## 5. Conclusions

In the study, esophageal/cardia cancer patients were selected as the research subjects to discuss the risk factors of postoperative arrhythmia and lung infection. Some patients were given targeted low-molecular anticoagulant drugs before surgery to explore the preventive effect of LMWH on the occurrence of DVT of the lower extremities in patients with esophageal/cardia cancer after surgery. The results found that age, preoperative disease history, hospital stay, and operation time were risk factors for postoperative adverse events in patients with esophageal/cardia cancer. The targeted anticoagulant LMWH can effectively reduce the incidence of DVT of lower extremities of patients with esophageal/cardia cancer. However, this study still has some shortcomings. This study has preliminary verified the prevention effects of targeted anticoagulant LMWH on the occurrence of DVT in patients with esophageal/cardia cancer after surgery and has not analyzed the molecular mechanism of its effects. In future work, we will further explore the specific mechanism of targeted anticoagulant LMWH in preventing lower extremity DVT in patients with esophageal/cardia cancer at the molecular and cellular levels. In conclusion, this study has clarified the risk factors for postoperative arrhythmia and lung infections. The targeted anticoagulant LMWH can prevent the occurrence of postoperative lower extremity DVT in patients with esophageal/cardia cancer. This provides an effective reference for the prognosis and prevention of esophagus/cardia cancer.

RETRACTED

## Figures and Tables

**Figure 1:** Comparison of risk factors for postoperative arrhythmia and normal groups. Note: *∗* means versus the normal group, *P* < 0.05; *∗∗* means versus the normal group, *P* < 0.01; and *∗∗∗* means versus the normal group, *P* < 0.001.

**Figure 2:** Comparison of related factors of postoperative lung infection: (a) comparison of age, blood loss, Alb, PLT, and BMI between the two groups of patients; (b) comparison of lymph node, hospital stay, operation time, FVC, and FEV1 between the two groups. Note: ^∗^ indicates versus the noninfection group, *P* < 0.05, and ^∗∗^ indicates versus the noninfection group, *P* < 0.01.

**Figure 3:** Comparison of risk factors for a postoperative lung infection. Note: ^∗∗^ indicates versus the noninfection group, *P* < 0.01, and ^∗∗∗^ indicates versus the noninfection group, *P* < 0.001.

**Figure 4:** Comparison of postoperative complications. A∼J in the abscissa represented anastomotic leakage, anastomotic stenosis, gastric stump fistula, thoracic-gastric syndrome, pulmonary complications, cardiovascular complications, gastric emptying disorder, respiratory failure, incision infection, and arrhythmia, respectively.

**Figure 5:** Comparison of preoperative complications between the two groups of patients.

**Figure 6:** Comparison of the proportion of patients with different surgical methods. 1∼5 in the abscissa represented left thoracic aortic arch gastroesophageal anastomosis; left thoracic aortic arch gastroesophageal anastomosis; left thoracic and neck two-incision gastroesophageal neck anastomosis; three-incision gastroesophageal neck anastomosis on the right chest, abdomen, and neck; and left chest and abdomen two-incision total gastrectomy and jejunal esophagus anastomosis.

RETRACTED

**Figure 7:** Comparison of surgical indicators: (a) comparison of anesthesia time and operation time and (b) comparison of intraoperative blood loss, intraoperative fluid replenishment, and postoperative drainage between the two groups.

**Figure 8:** Comparison of the incidence of DVT in lower extremities between the two groups.

**Figure 9:** Ultrasound image of the veins of the lower extremities: (a∼c) normal lower extremity vein ultrasound images and (d∼f) postoperative lower extremity vein ultrasound images.

**Figure 10:** Risk assessment scale of the lower extremity DVT between the two groups of patients in different periods. Note: *∗* indicates versus the control group, *P* < 0.05; *∗∗* indicates versus the control group, *P* < 0.01; and  ^*∗∗∗*^ indicates versus the control group, *P* < 0.001.

**Figure 11:** Comparison of D-dimer values between the two groups of patients in different periods. Note: ^∗^ indicates versus the control group, *P* < 0.05, and ^∗∗^ indicates versus the control group, *P* < 0.01.

**Table 1:** Logistic regression of risk factors for arrhythmia.

Risk factors	Regression coefficients	Standard error	OR	95% CI	*P* value
Age ≥65 years old	2.825	1.314	2.254	1.035, 5.428	0.009
Abnormal preoperative ECG	1.128	0.517	3.029	0.219, 2.095	0.021
CHD before surgery	1.006	0.428	2.751	0.528, 1.627	0.001
COPD before surgery	0.985	0.526	5.857	0.131, 1.825	0.008
Operation time ≥4h	0.829	0.617	4.988	0.122, 1.956	0.007
Preoperative serum potassium <4.0	0.622	0.261	1.484	0.076, 1.083	0.028

**Table 2:** Logistic regression of risk factors for a postoperative lung infection.

Risk factors	Regression coefficients	Standard error	OR	95% CI	*P* value
Age	0.185	0.094	1.189	1.049, 1.653	0.027
Diabetes before surgery	0.822	0.326	2.022	1.157, 3.629	0.018
COPD before surgery	1.363	0.317	3.394	2.018, 6.671	0.001
The hospital stay	0.784	0.239	2.176	1.351, 3.438	0.001
FEV1	−5.176	1.983	0.398	4.325, 15.082	0.002

**Table 3:** Comparison of basic data of the two groups of patients.

Group	Control group (*N* = 62)	Anticoagulant group (*n* = 33)	*t* value or *χ*^2^ value	*P* value
Age (years)	61.14 ± 3.44	60.88 ± 3.39	1.782	0.206
Female (cases, (%))	12 (27.27)	11 (28.94)	2.421	0.253
Male (cases, (%))	32 (72.73)	27 (70.05)		
BMI (kg/m^2^)	23.87 ± 3.32	21.25 ± 3.19	3.301	0.021
Tumor site				
Esophagus (cases, (%))	29 (65.91)	25 (65.78)	1.283	0.313
Cardia (cases, (%))	15 (34.09)	13 (34.21)		
Pathological types				
Squamous cell carcinoma	30 (68.18)	25 (65.79)	6.254	0.306
Adenocarcinoma	14 (31.82)	13 (34.21)		

RETRACTED

## Data Availability

The data used to support the findings of this study are available from the corresponding author upon reasonable request.
